This article has been retracted.

# Effects of Circ_0109046 Regulating Mir-338-3p on the Malignant Behavior of A2780 Cells

**DOI:** 10.1155/2022/4655939

**Published:** 2022-09-20

**Authors:** Yue Zhao, Haidan Diao, Jiangning Li, Xin Guan, Xiaofang Tian, Wei Guo, Baoxi Zhang, Dan Hao, Jian Yang

**Affiliations:** The Third People's Hospital of Da Lian, Dalian 116600, China

## Abstract

**Objective:**

The objective is to explore the action and mechanism of circ_0109046 on the malignant phenotypes of ovarian cancer cells.

**Methods:**

Circ_0109046 and miR-338-3p expression were detected by quantitative real-time polymerase chain reaction (qRT-PCR). In vitro assays were conducted to investigate the action of circ_0109046 and miR-338-3p on ovarian cancer cell growth and metastasis. Western blotting was utilized to investigate the contents of apoptosis-related markers. The binding between circ_0109046 and miR-338-3p was validated using dual-luciferase reporter assay.

**Results:**

Circ_0109046 was increased, while miR-338-3p content was decreased in ovarian cancer tissues. Deficiency of circ_0109046 or the upregulation of miR-338-3p was observed to weaken cell proliferative, migratory, and invasive abilities and elevated cell apoptosis rate in ovarian cancer. Circ_0109046 targetedly suppressed miR-338-3p. Down-regulation of miR-338-3p was able to reverse the repressing impacts of circ_0109046 silencing on ovarian cancer growth and mobility.

**Conclusion:**

Circ_0109046 silencing impaired the proliferation, migration, and invasion of ovarian cancer cells through negatively regulating miR-338-3p in vitro, indicating the potential implication of circ_0109046 in ovarian cancer progression.

## 1. Introduction

Ovarian cancer is a common malignant tumor affecting women's life, health, and safety. Its pathogenesis is still unclear, and there is a lack of effective treatment [1]. Therefore, it is of great significance to find effective therapeutic targets to prevent ovarian cancer.

Circular RNA (circRNA) is a kind of noncoding RNA, which is highly stable due to its closed structure. A vast array of abnormally expressed circRNAs, such as circ_0005276 [2], circ_0004390 [3], and circPIP5K1A [4], have been discovered in ovarian cancer, which are closely related to the clinicopathological features and prognosis of ovarian cancer patients; moreover, functional experiments further confirmed their involvement in the tumorigenesis of ovarian cancer, implying that circRNAs may be promising candidates for the development of ovarian cancer therapeutic method. Recently, research showed that circ_0109046 was highly expressed in endometrial cancer and predicted poor prognosis; functionally, circ_0109046 lack inhibited the proliferation and invasiveness of endometrial cancer cells by miR-105 [5]. However, the action and mechanism of circ_0109046 on the ovarian cancer cell malignant phenotypes remain vague. MicroRNA (miRNA) is also a kind of noncoding RNA, and circRNA can act as a sponge for miRNA to affect the malignant progression of cancer cells [6]. In our study, preliminary online prediction revealed that circ_0109046 has complementary sequences of miR-338-3p. A previous study showed the decreased miR-338-3p in ovarian cancer, which was related to the bad survival rate [7]. However, the effect of miR-338-3p and the relationship between circ_0109046 and miR-338-3p are also unknown yet.

This study used the A2780 cells to explore the functions of circ_0109046 and miR-338-3p on ovarian cancer cell malignant phenotypes and further investigated whether circ_0109046 could exert its effects by miR-338-3p in ovarian cancer.

## 2. Materials and Methods

### 2.1. Patient Samples

A total of 57 patients (45.26 ± 6.59 years) with ovarian cancer who were hospitalized in our hospital from May 2017 to May 2020 were selected as the research objects. During the operation, the cancer tissues and adjacent normal tissues of the patients were collected and then stored in liquid nitrogen. Inclusion criteria are confirmed by pathological diagnosis for the first time. Exclusion criteria are preoperative radiotherapy, chemotherapy, and other treatments, combined with other malignant tumors. The study was approved by the ethics committee of our hospital in accordance with the Declaration of Helsinki, and all patients provided written consent forms.

### 2.2. Cell Culture

A2780 cells were purchased from Shanghai Cell Bank, Chinese Academy of Sciences (Shanghai, China), and then grew in RPMI-1640 medium (Solarbio, Beijing, China) supplemented with 10% fetal bovine serum (FBS), 100 U/mL of penicillin, and 100 *μ*g/mL of streptomycin (Solarbio) with 5% CO_2_ at 37°C.

### 2.3. Cell Transfection

The short hairpin RNA (shRNA) against circ_0109046 (sh-circ_0109046), miR-338-3p mimic (miR-338-3p), or inhibitor (anti-miR-338-3p) and negative control (sh-NC, miR-NC, or anti-NC) were obtained from Sangon Biotech (Shanghai, China). Cell transfection was carried out with reference to the Lipofectamine 2000 kit (Invitrogen, Camarillo, CA, USA) with 2.5 mL A2780 cells (5.0 × 104/mL). 24 h later, the expression of circ_0109046 or miR-338-3p was detected in the A2780 cells to verify the transfection efficiency.

### 2.4. Quantitative Real-Time Polymerase Chain Reaction (qRT-PCR)

Total RNA was prepared using the RNeasy Mini Kit as per the protocol (Qiagen, Crawley, UK). Thereafter, the obtained RNAs were subjected to reverse-transcription to synthesize cDNA using the PrimeScript RT polymerase (Takara, Otsu, Japan), and then qRT-PCR was performed by SYBR real-time PCR mixture (Takara). The conditions were programmed as follows: 42°C 5 min, 95°C 10 s, followed by 40 cycles at 95°C for 5 s, and 60°C 30 s. The gene expression was processed using the 2^−ΔΔCt^ method, and U6 or glyceraldehyde-3-phosphate dehydrogenase (GAPDH) was used as the control. The primers for qRT-PCR are listed in Table 1.

### 2.5. Cell Counting Kit-8 (CCK-8) Assay

Transfected A2780 cells (5.0 × 10^4^ cells/mL) were seeded into a 96-well plate and cultured for 24 h, followed by reacting with CCK-8 solution (10 *μ*L, Beyotime, Shanghai, China) for another 2 h. Then, the optical density values at 450 nm were measured.

### 2.6. Flow Cytometry

After transfection, 2.5 mL A2780 cells of each group (5.0×104 cells/mL) were collected and resuspended in 500 *μ*L binding buffer (1×). Then, cell apoptosis was analyzed by flow cytometry after staining orderly with 10 *μ*L Annexin V-fluorescein isothiocyanate (FITC) and 5 *μ*L propidium iodide (PI) (Life Technologies, Scotland, UK).

### 2.7. Transwell Assay

After transfection, 100 *μ*L A2780 cells (5.0 × 10^4^/mL) in each group suspended in serum-free medium were added to the top chambers of 24-well Transwell chambers (Corning, Cambridge, MA, USA) that were precoated without (for migration) or with Matrigel (Solarbio) (for invasion), and 500 *μ*L of serum-containing medium was added to the lower chamber for 24 h culture. Finally, migrated and invaded cells were observed and counted by a microscope (Bio-Rad, Hercules, CA, USA) after crystal violet staining for 30 min.

### 2.8. Western Blotting

A2780 cells in each group were split by RIPA reagent (Yeasen, Shanghai, China) for 30 min on ice. Equal amounts of samples (20 *μ*g) were separated by 10% SDS-PAGE and then electrophoretically shifted onto PVDF membranes, followed by blocking with 5% skim milk powder for 2 h. The membranes were interacted with primary antibodies against B-cell lymphoma-2 (Bcl-2) (1 : 2000, ab182858, Abcam, Cambridge, MA, USA) and BCL2-associated X (Bax) (1 : 1000, ab32503, Abcam) and GAPDH (1 : 5000 m ab8245, Abcam) all night at 4°C. Following secondary incubation at 37°C for 1 h, protein signals were quantified by an ECL reagent (Beyotime).

### 2.9. Dual-Luciferase Reporter Assay

The fragments of circ_0109046 carrying the wild-type (WT) binding site of miR-338-3p or mutated (MUT) sequences were cloned into pmirGLO vectors (Solarbio) to establish luciferase reporter vectors (WT/MUT-circ_0109046), which were then transfected into A2780 cells together with miR-NC or miR-338-3p mimics, and the luciferase activity in each group was tested 48 h later by dual-luciferase reporter kit (Solarbio).

### 2.10. Statistical Analysis

The experimental results were expressed as mean ± standard deviation (SD). SPSS 22.0 software was used for statistical analysis. The *t*-test was used for group comparison. *P* < 0.05 indicated statistically significant.

## 3. Results

### 3.1. The Expression of Circ_0109046 and MiR-338-3p in Ovarian Cancer

As shown in Figure 1(a), circ_0109046 expression was higher in ovarian cancer tissues (II) than those in adjacent normal tissues (I). However, miR-338-3p expression was opposite that was lowly expressed in ovarian cancer tissues (II) (Figure 1(b)).

### 3.2. Effects of Circ_0109046 on Ovarian Cancer Cell Malignant Phenotypes

As shown in Table 2, deficiency of circ_0109046 suppressed A2780 cell proliferation, migration, and invasion compared with the sh-NC group. Besides, circ_0109046 silencing induced apoptosis in A2780 cells relative to sh-NC transfection, evidenced by increased apoptosis rate and Bcl-2 expression, as well as decreased Bax expression (Table 2 and Figures 2(a) and 2(b)).

### 3.3. Circ_0109046 Acted as a Sponge for MiR-338-3p

According to the prediction of CircInteractome, circ_0109046 possesses the binding site of miR-338-3p (Figure 3(a)). Furthermore, miR-338-3p mimic was found to reduce the luciferase activity of WT-circ_0109046 group in A2780 cells, but not the MUT-circ_0109046 group compared with the control group (Figure 3(b)). Besides, sh-circ_0109046 transfection in A2780 cells led to an increase of miR-338-3p expression level (Figure 3(c)).

### 3.4. Effects of MiR-338-3p on Ovarian Cancer Cell Malignant Phenotypes

As shown in Table 3 and Figures 4(a) and 4(b), miR-338-3p elevation impaired A2780 cell proliferation, migration, and invasion but evoked cell apoptosis compared with the miR-NC groups; besides, miR-338-3p overexpression decreased Bcl-2 expression as well as increased Bax expression in A2780 cells.

### 3.5. MiR-338-3p Inhibition Abolished the Effects of Circ_0109046 Knockdown on Ovarian Cancer Cell Malignant Phenotypes

As exhibited in Table 4 and Figures 5(a) and 5(b), down-regulation of miR-338-3p expression could attenuate circ_0109046 knockdown-mediated inhibition of cell proliferative, migratory, and invasive abilities, as well as the promotion of cell apoptotic rate in A2780 cells.

## 4. Discussion

CircRNAs exist widely in eukaryotes, and the circRNA/miRNA axis has been shown to be implicated in regulating the malignant behaviors of tumor cells that has an important impact on the genesis and progression of malignancies [8]. Studies have shown a variety of circRNAs in modulating ovarian cancer cell malignant behaviors. For instance, circ_0026123 silencing could inhibit the proliferative and migratory capacities of ovarian cancer cells by miR-124-3p/Enhancer of zeste homolog 2 (EZH2) axis, thereby inhibiting tumor malignant process [9]. An up-regulated circ_0007841 was discovered in ovarian cancer, and circ_0007841 enhanced cancer cell metastasis and growth *in vitro* and in nude mice by up-regulating Mex-3 RNA Binding Family Member C expression through competitively adsorbing miR-151-3p, indicating an oncogenic role of circ_0007841 in ovarian cancer [10]. Besides, upregulation of circ_0007874 inhibited the migration and proliferation of ovarian cancer cells by competitively adsorbing miR-760 and up-regulating suppressor of cytokine signaling 3 (SOCS3) expression [11]. Circ_0109046 is a stable circRNA, while the effects and mechanism of circ_0109046 on ovarian cancer have not been elucidated. In this study, circ_0109046 was showed to be increased in ovarian cancer, suggesting the potential promoting action of it in the development of ovarian cancer. Functionally, reduction of circ_0109046 reduced the proliferative, migratory, and invasive abilities of A2780 cells and at the same time promoted apoptosis by enhancing the content of pro-apoptotic Bax protein and declining the level of anti-apoptotic Bcl-2 protein, indicating that circ_0109046 lack inhibited the malignant progression of ovarian cancer cells *in vitro*. Subsequently, we further elucidated by which knockdown of circ_0109046 hindered the malignant biological behaviors of ovarian cancer cells, and we identified the circ_0109046/miR-338-3p axis in cancer cells.

MiR-338-3p has been found to be abnormally expressed in various cancers and involved in cancer development. For example, down-regulation of miR-338-3p expression expedited the proliferation of lung cancer cells *in vitro* and *in vivo* [12]. MiR-338-3p upregulation could hinder hepatocellular carcinoma cell metastasis by targeting Zinc Finger E-Box Binding Homeobox 2 (ZEB2) [13]. A decreased miR-338-3p was found in clear cell renal cell carcinoma, which resulted in the promotion of cancer cell proliferation, migration, and invasiveness through targetedly inhibiting ETS Proto-Oncogene 1, Transcription Factor (ETS1) expression [14]. In addition, miR-338-3p was also declined in glioblastoma [15] and pancreatic cancer [16] and performed anticancer action to affect the development of these tumors. Importantly, miR-338-3p also had anti-growth and anti-metastasis effects on ovarian cancer cells [17]. Consistent with previous findings, this study also showed a lowly expressed miR-338-3p in ovarian cancer. Functionally, upregulation of miR-338-3p was found to reduce the mobility and growth in A2780 cells. At the same time, we also found that miR-338-3p deficiency reduced the suppressive effects of circ_0109046 lack on ovarian cancer cells, further suggesting that circ_0109046 affected ovarian cancer tumorigenesis by miR-338-3p.

In conclusion, knockdown of circ_0109046 or upregulation of miR-338-3p significantly impaired the mobility and growth of ovarian cancer cells. Mechanistically, miR-338-3p was targeted by circ_0109046; circ_0109046 performed its carcinogenic effects via targeting miR-338-3p, implying new targets for the treatment of ovarian cancer.

## Figures and Tables

**Figure 1:** The expression of circ_0109046 and miR-338-3p in ovarian cancer. (a-b) The expression of circ_0109046 and miR-338-3p in ovarian cancer tissues and adjacent normal tissues detected by qRT-PCR. Note. (I) adjacent normal tissues; (II) ovarian cancer tissue. ^*∗*^*P* < 0.05.

**Figure 2:** Effects of circ_0109046 on ovarian cancer cell apoptosis. (a) Flow cytometry for A2780 cell apoptosis after circ_0109046 knockdown. (b) Western blotting for the levels of Bax and Bcl-2 in A2780 cells after circ_0109046 knockdown. ^*∗*^*P* < 0.05.

**Figure 3:** Circ_0109046 acted as a sponge for miR-338-3p. (a) The potential binding sites between circ_0109046 and miR-338-3p. (b) The interaction analysis by dual-luciferase reporter assay. (c) Increased miR-338-3p level in A2780 cells after circ_0109046 knockdown. ^*∗*^*P* < 0.05 compared with miR-NC group; ^#^*P* < 0.05 compared with sh-NC group.

**Figure 4:** Effects of miR-338-3p on ovarian cancer cell apoptosis. (a) Flow cytometry for A2780 cell apoptosis after miR-338-3p overexpression. (b) Levels of Bax and Bcl-2 in A2780 cells after miR-338-3p overexpression by western blotting. ^*∗*^*P* < 0.05.

**Figure 5:** Effects of circ_0109046/miR-338-3p on ovarian cancer cell apoptosis. After co-transfection of sh-circ_0109046 and anti-miR-338-3p, (a) flow cytometry for A2780 cell apoptosis; (b) levels of apoptosis-related markers in A2780 cells by western blotting. ^*∗*^*P* < 0.05.

**Table 1:** The primers for qRT-PCR.

Name	Forward	Reverse
circ_0109046	5′-TCTTCCAGACACGATTCCGC-3′	5′-AGGGGAGGGATAGCACACAT-3′
GAPDH	5′-GTCTCCTCTGACTTCAACAGCG-3′	5′-ACCACCCTGTTGCTGTAGCCAA-3′
miR-338-3p	5′-GCCGAGTCCAGCATCAGTGAT-3′	5′-CAGTGCGTGTCGTGGAGT-3′
U6	5′-CTCGCTTCGGCAGCACATATA-3′	5′-AACGCTTCACGAATTTGCGT-3′

**Table 2:** Effects of circ_0109046 knockdown on A2780 cell proliferation, apoptosis, migration, and invasion ($\bar{x}$ ± *s*, *n* = 9).

Groups	Circ_0109046	%		Cells		Bax	Bcl-2
		Proliferation	Apoptosis	Migration	Invasion		
Sh-NC	1.00 ± 0.00	0.00 ± 0.00	7.61 ± 0.48	161.56 ± 9.83	218.11 ± 11.62	0.20 ± 0.06	0.76 ± 0.06
Sh-circ_0109046	0.41 ± 0.05^*∗*^	49.01 ± 3.32^*∗*^	21.60 ± 1.20^*∗*^	82.00 ± 4.81^*∗*^	114.11 ± 6.35^*∗*^	0.64 ± 0.05^*∗*^	0.32 ± 0.04^*∗*^
*t*	35.400	44.286	32.473	21.810	23.562	16.901	18.305
*P*	0.000	0.000	0.000	0.000	0.000	0.000	0.000

**Table 3:** Effects of miR-338-3p overexpression on A2780 cell proliferation, apoptosis, migration, and invasion ($\bar{x}$ ± *s*, *n* = 9).

Groups	miR-338-3p	%		Cells		Bax	Bcl-2
		Proliferation	Apoptosis	Migration	Invasion		
miR-NC	1.00 ± 0.00	0.00 ± 0.00	7.67 ± 0.72	162.89 ± 12.47	212.56 ± 14.70	0.21 ± 0.02	0.74 ± 0.08
miR-338-3p	3.20 ± 0.09^*∗*^	54.77 ± 3.75^*∗*^	23.00 ± 1.54^*∗*^	65.78 ± 4.31^*∗*^	92.11 ± 4.15^*∗*^	0.72 ± 0.06^*∗*^	0.25 ± 0.02^*∗*^
*t*	73.333	43.816	27.053	22.081	23.657	24.191	17.826
*P*	0.000	0.000	0.000	0.000	0.000	0.000	0.000

**Table 4:** Effects of circ_0109046/miR-338-3p on A2780 cell proliferation, apoptosis, migration, and invasion ($\bar{x}$ ±*s* , *n* = 9).

Groups	miR-338-3p	%		Bax	Bcl-2	Cells	
		Proliferation	Apoptosis			Migration	Invasion
Sh-circ_0109046 + anti-miR-NC	1.00 ± 0.00	49.24 ± 3.31	21.38 ± 1.17	0.63 ± 0.06	0.30 ± 0.04	78.89 ± 5.38	114.67 ± 5.87
Sh-circ_0109046 + anti-miR-338-3p	0.39 ± 0.05^*∗*^	22.34 ± 0.81^*∗*^	12.32 ± 0.65^*∗*^	0.35 ± 0.03^*∗*^	0.59 ± 0.05^*∗*^	143.67 ± 9.51^*∗*^	183.00 ± 10.54^*∗*^
*t*	36.600	23.682	20.307	12.522	13.587	17.786	16.991
*P*	0.000	0.000	0.000	0.000	0.000	0.000	0.000

## Data Availability

The labeled dataset used to support the findings of this study is available from the corresponding author upon request.
